The article "Mechanism of Zuogui pill enhancing ovarian function and skin elastic repair in premature aging rats based on artificial intelligence medical image analysis" was retracted in 2025. Reasons: compromised peer review; a compromised editor; unreliable results or conclusions; concerns about the results or conclusions.

# Mechanism of Zuogui pill enhancing ovarian function and skin elastic repair in premature aging rats based on artificial intelligence medical image analysis

**DOI:** 10.1111/srt.70050

**Published:** 2024-09-09

**Authors:** Xinpei Zhang, Fuju Wang, Xiaodan Zhu, Lan Xu, Ling Qin, Wenjuan Xu, Bozhen Fan

**Affiliations:** ^1^ Department of Obstetrics and Gynecology Putuo Hospital, Shanghai University of Traditional Chinese Medicine Shanghai China; ^2^ Department of Gynecology of Traditional Chinese Medicine Putuo Hospital, Shanghai University of Traditional Chinese Medicine Shanghai China

**Keywords:** artificial intelligence, elastic skin repair, medical image analysis, ovarian function, premature aging rats, Zuogui Wan

## Abstract

**Background:**

AI medical image analysis shows potential applications in research on premature aging and skin. The purpose of this study was to explore the mechanism of the Zuogui pill based on artificial intelligence medical image analysis on ovarian function enhancement and skin elasticity repair in rats with premature aging.

**Materials and Methods:**

The premature aging rat model was established by using an experimental animal model. Then Zuogui pills were injected into the rats with premature aging, and the images were detected by an optical microscope. Then, through the analysis of artificial intelligence medical images, the image data is analyzed to evaluate the indicators of ovarian function.

**Results:**

Through optical microscope image detection, we observed that the Zuogui pill played an active role in repairing ovarian tissue structure and increasing the number of follicles in mice, and Zuogui pill also significantly increased the level of progesterone in the blood of mice.

**Conclusion:**

Most of the ZGP‐induced outcomes are significantly dose‐dependent.

## 1 INTRODUCTION

Premature aging is a widespread and concerned health problem. With the increasing trend of population aging, premature aging has a serious impact on human physical and mental health. Premature aging is often accompanied by problems such as decreased ovarian function and decreased skin elasticity, which have a great adverse impact on the quality of life of patients. In the past few decades, artificial intelligence technology has made great progress in the field of medicine. In particular, artificial intelligence medical image analysis provides a new way to understand and diagnose diseases. The image data of rat ovaries and skin obtained by high‐resolution imaging equipment and analyzed by advanced artificial intelligence algorithms can quantify and identify relevant indicators, providing more comprehensive information for the research and treatment of premature aging. The loss of skin elasticity can lead to problems such as wrinkles, sagging skin, and reduced elasticity, further exacerbating the symptoms of premature aging in patients. Premature ovarian insufficiency (POI) featured with menstrual disturbance with heightened gonadotrophins and depressed estradiol. The prevalence is about 1% but there has become a gradual increase in the occurrence. Women with POI have less chance to gestate spontaneously. Untreated patients are associated to a reduced life span, mainly owing to cardiovascular disease.^1^, ^2^ POI is a heterogeneous and multifactorial syndrome, primarily related to chromosome, gene, and autoimmune, followed by iatrogenicity, surgery, toxicity of chemoradiotherapy, and infection. The etiology is still unknown in 60%–70% of cases.^3^

The article "Mechanism of Zuogui pill enhancing ovarian function and skin elastic repair in premature aging rats based on artificial intelligence medical image analysis" was retracted in 2025. Reasons: compromised peer review; a compromised editor; unreliable results or conclusions; concerns about the results or conclusions.

Primordial follicles are formed early in life and remain latent for lengthy periods in mammals. Primordial follicle activation (PFA) ushers in the recommencement of growth. PFA and subsequent follicle development are unalterable, and initiated follicles will undergo atresia if not chosen to advance. Therefore, it is of great value to study the regulatory channels and mechanisms of PFA for POI.^4^ Strong correlation exists between DNA repair and damage in ovarian granulosa cells (GCs) and POI.^5^, ^6^ Therefore, an exploration of how pathways regulate primordial follicle maintenance is required to elaborate the POI.

Traditional Chinese medicine (TCM) states that “kidney governing reproduction,” and oocytes derive from kidney essence.^7^ Therefore, the underlying pathogenesis of POI is associated with kidney essence shortage. POI treatment with Chinese medicine produces better outcomes.^8^ Zuogui pill (ZGP), a TCM effective in tonifing kidney essence and made up of *Rehmanniae Radix Praeparata*, *Corni Fructus*, and *Dioscoreae Rhizoma*, *etc*., can strengthen the kidney, produce essence, and improve the marrow.^9^ However, the mechanism of ZGP improving POI is complicated and still unclear.

Optical microscope image detection is the detection method that uses optical microscope to observe and analyze samples. By zooming in on the structure of cells and tissues, it can provide high‐resolution images, allowing researchers to observe and analyze cells and tissues in detail. In the study of the mechanism of premature aging, optical microscope image detection has many advantages and application potential. Optical microscopy image inspection is a non‐invasive method that does not require the destruction or damage of the sample, so the integrity and viability of the sample can be maintained. This is important for studying changes in ovarian function because the mechanisms of premature aging involve alterations at the cellular and tissue levels. By using optical microscope image detection, researchers can observe and analyze the structure of ovarian tissue, as well as the associated networks of cells and blood vessels. Optical microscopy image detection can extract important biological characteristics, such as the number, size, and development of follicles. These features are critical for assessing the status of ovarian function and the extent of premature aging. Through quantitative analysis of the images, objective, repeatable data can be obtained and compared with healthy groups. This will help to reveal the mechanism of premature aging and provide an important reference index for the diagnosis and treatment of premature aging. Optical microscope image detection technology can also be combined with other methods and techniques for comprehensive analysis. For example, specific biomarkers can be labeled and detected in combination with fluorescent staining techniques to more precisely assess ovarian function and cell activity. It can also be combined with molecular biological techniques, such as gene expression analysis or protein quantification, to reveal the underlying molecular mechanisms of premature aging. Therefore, optical microscope image detection has important application potential in studying the mechanism of premature aging. It can provide high‐resolution images, observe and analyze the structure and characteristics of ovarian tissue, and provide important clues for understanding the mechanism of premature aging. Through the application of optical microscope image detection, the change process of premature aging is more deeply understood, and the scientific basis for the prevention and treatment of premature aging is provided.

The article "Mechanism of Zuogui pill enhancing ovarian function and skin elastic repair in premature aging rats based on artificial intelligence medical image analysis" was retracted in 2025. Reasons: compromised peer review; a compromised editor; unreliable results or conclusions; concerns about the results or conclusions.

In our work, the protective effect of different doses of ZGP on POI was revealed through a rat model, and whether ZGP improved POI through PI3K/Akt/mTOR signaling pathway was discussed. The findings also proved ZGP an effective choice for POI. At present, the research on artificial intelligence medical image analysis and skin elastic repair is still relatively limited. There is a lack of understanding of the mechanisms of ovarian function and skin elastic repair in premature aging rats. By combining artificial intelligence medical image analysis with skin elastic repair, this study will provide new insights into the mechanisms of ovarian function and skin elastic repair in premature aging rats, and provide new ideas for the future development of effective means to treat premature aging. This will help improve the quality of life of patients with premature aging and provide scientific support to address the challenges posed by an aging population.

## 2 METHODS

### 2.1 Animal

Twenty‐five healthy 5‐week‐old female Wistar rats weighing 200 ± 20 g. Rats were placed in a specific pathogen‐free, biosecurity‐protected animal laboratory with a temperature of 20−24°C, humidity of 50%−60%, and an artificial light/dark cycle of 12 h, supplied with rat cubes and tap water ad libitum. The experiment moved into the next phase after rats had undergone 7 days of adaptive feeding. All animal experiments conducted in this study adhered to the guiding principles outlined in the comprehensive document known as the “Guide for the Care and Use of Laboratory Animals.” This meticulous approach ensured that the welfare and ethical considerations pertaining to the animals involved were given the utmost attention and care. By following the guidelines outlined in this guide, the researchers responsible for this study demonstrated their commitment to upholding the highest standards of animal welfare and scientific integrity. The principles emphasized in this guide encompassed various aspects, including the appropriate housing, husbandry, and care of the laboratory animals, as well as the meticulous planning and execution of the experiments. The researchers took great care to ensure that the animals' well‐being was prioritized throughout the entire experimental process. This included providing the animals with suitable environments, proper veterinary care, and minimizing any potential distress or discomfort. Additionally, the researchers made sure to obtain the necessary ethical approvals before commencing the experiments, further attesting to their commitment to conducting responsible and humane research (NIH publication No. 85‐23, revised 1996).

### 2.2 Drug preparation and instruments

Cisplatin was obtained from Sigma‐Aldrich (St. Louis, MO), while ZGP was acquired from Shanghai Leiyun Shangfengbang Pharmaceutical Co., Ltd. For the intragastric administration, we designed three different dose levels: low, moderate, and high. We procured the necessary kits for the detection of malondialdehyde (MDA) and superoxide dismutase (SOD) from a reputable supplier called Shanghai Enzyme Biotechnology Co., Ltd. These detection kits, specifically designed and developed by the company, are widely recognized for their accuracy and reliability in measuring the levels of MDA and SOD. The ELISA technique, utilizing these kits, allows for precise and sensitive quantification of the targeted biomarkers in biological samples. Shanghai Enzyme Biotechnology Co., Ltd. has a strong reputation in the field of biotechnology and is known for providing high‐quality products that meet the stringent requirements of scientific research. By utilizing their detection kits, we ensured that the measurement of MDA and SOD in our study was performed with high precision and consistency. The ELISA process, facilitated by these kits, enabled us to analyze and quantify the enzymatic activity levels accurately, contributing to the robustness and validity of our experimental results. It is important to note that the source of these kits, Shanghai Enzyme Biotechnology Co., Ltd. was chosen based on their expertise and reputation in providing reliable and well‐validated kits for scientific research purposes. Beyotime Biotechnology provided us with the protease inhibitor phenylmethylsulfonyl fluoride (PMSF), radio‐immunoprecipitation assay (RIPA), and the enhanced chemiluminescence (ECL) reagent kit. The TUNEL assay enables the visualization and quantification of DNA fragmentation, a hallmark of apoptotic cell death. The ApopTag Peroxidase in situ apoptosis detection kit, specifically designed by Chemicon International, incorporates a series of carefully optimized and validated reagents and protocols. These components work together synergistically to ensure accurate and specific labeling of apoptotic cells within tissue samples. Through the TUNEL procedure, the TdT enzyme adds dUTP‐biotin labeled nucleotides to the 3′‐OH ends of fragmented DNA. Subsequently, the incorporated biotin labels are detected using peroxidase‐conjugated streptavidin, which produces a localized color reaction at the site of apoptotic cells. This distinctive staining enables the precise identification of apoptotic cells within the tissue sections, facilitating their quantitative analysis. Chemicon International, as a reputable provider of apoptosis detection kits and related products, is widely acknowledged for its commitment to quality and reliability. By utilizing their ApopTag Peroxidase in situ apoptosis detection kit, we ensured that our study benefited from validated and standardized methodologies, minimizing potential sources of variability and enhancing the accuracy of our apoptotic cell quantification. We obtained the primary antibodies, PI3K (4249), Akt (4691), and mTOR (2983) from Cell Signaling Technology, while p‐PI3K (ab182651), p‐Akt (ab38449), p‐mTOR (ab84400), Bcl‐2 (ab59348), Bcl‐2‐Associated X (Bax) (ab32503), cysteinyl aspartate‐specific proteinase (Caspase)‐3 (ab184787) and β‐actin (ab8226) were acquired from Abcam. EarthOx Life Sciences provided the goat anti‐rabbit secondary antibodies.

The article "Mechanism of Zuogui pill enhancing ovarian function and skin elastic repair in premature aging rats based on artificial intelligence medical image analysis" was retracted in 2025. Reasons: compromised peer review; a compromised editor; unreliable results or conclusions; concerns about the results or conclusions.

### 2.3 Experimental protocol

Rats were divided into two groups at random: blank (group A, *n* = 5) and modeling (*n* = 20), then split into squirrel cages for observation according to the grouping. To establish the POI model, the modeling group was intraperitoneally injected with 4 mg/kg cisplatin on the 1st and 8th days. The blank group was injected with an identical saline in volume. The dosage would be adjusted each week in line with the weight alteration.

Vaginal smears were collected every morning to monitor rat's estrus cycle. A normal estrous cycle presents as a cycle of 4–5 days and the estrus period, pre‐estrus, estrus, and late‐estrus appeared in turn, while abnormality manifesting as continuous estrus, a prolonged estrus cycle of 6–10 days, or absence of pre‐estrus and estrus, demonstrate successful modeling. POI was evaluated using the following inclusion criteria: alterations in mental and functional status, such as decreased calorie and fluid intake, sluggish responses, decreased locomotion, and vaginal epithelial exfoliative cell smears demonstrating an estrous cycle abnormality as well. It was defined as exclusion criteria in case of vaginal epithelial cytology smears demonstrating a normal estrous cycle, regardless of alterations in mental and active status.

Drug‐induced POI rats were classified into four groups at random: groups B (*n* = 5), the model control group, and three ZGP groups (group C‐E, the low, moderate, and high‐dose group respectively, *n* = 5/group). The ZGP groups received daily intragastric administration (i.g.) of ZGP solution at a concentration of 0.2 g/mL for 42 days. The low ZGP group was administered at a dosage of 0.8 g/kg, the moderate ZGP group at a dosage of 1.6 g/kg, and the high ZGP group at a dosage of 3.2 g/kg. On the other hand, rats in the control groups were injected with 2 mL of saline solution.

Rats’ blood samples from the orbital venous plexus were gathered on non‐estrus period under anesthesia through intraperitoneal injection of 10% chlorali hydras (3 mL/kg) on day 70, as well as oophorectomy. Subsequently, euthanasia was implemented via cervical dislocation. The blood samples were coagulated at room temperature for roughly 1 h, after which serum was acquired by centrifuging for 20 min at 3000 rpm/min and then kept at −80°C. Some ovarian tissue was soaked in 10% formaldehyde for histopathology, while the remaining was frozen at −80°C for protein testing.

Serum concentrations of MDA and SOD were measured by ELISA. Operations were performed strictly complied with the manufacturers’ protocols.

### 2.4 Immunohistochemistry (IHC)

After the surgical removal of the ovaries, meticulous procedures were followed to ensure their optimal preservation and preparation for subsequent analyses. Specifically, half of the excised ovaries were immersed in a 4% paraformaldehyde solution at room temperature for a duration of 24 h. This paraformaldehyde fixation process served to stabilize the ovarian tissue and prevent degradation or damage to the cellular components. Following the fixation step, the ovaries underwent a series of preparation procedures to facilitate their subsequent histological examination. Firstly, the fixed tissues were subjected to dehydration using a gradually increasing series of ethanol concentrations. This step involved immersion of the specimens in solutions of ascending ethanol concentrations, facilitating the gradual removal of water from the tissue while maintaining their structural integrity. Subsequently, the dehydrated specimens were cleaned using xylene, a solvent commonly employed in histology procedures for effective removal of the dehydrating agent and facilitating subsequent embedding. The use of xylene helped in clearing the tissues and preparing them for embedding in paraffin wax, a widely used embedding medium due to its compatibility with subsequent sectioning processes. To facilitate the preparation of ovarian slices suitable for immunohistochemistry (IHC) analysis, the paraffin‐embedded tissues were cut into sections of approximately 4 μm thickness. These thin sections were carefully excised using specialized microtome equipment and mounted onto glass slides for further analysis. The resulting tissue sections were then subjected to a series of steps to optimize their suitability for immunohistochemical staining. To ensure proper section adherence and eliminate any potential artifacts, the slides with ovarian sections were incubated at a controlled temperature of 60°C for 1 h, allowing the tissue sections to firmly attach to the glass slides. Following this, the slides underwent a process known as deparaffinization, which involved treating the sections with xylene to remove the paraffin wax. Graduated ethanol solutions were then used to rehydrate the tissue sections, gradually replacing the xylene with increasing concentrations of ethanol. Furthermore, to enhance the detectability of target antigens within the ovarian tissue sections during immunohistochemistry, an antigen retrieval step was performed. This involved subjecting the slides to high microwave temperature using a sodium citrate buffer (pH 6.0) for 30 min. The purpose of this step was to restore the accessibility and immunoreactivity of the antigens within the tissue sections, which might have been altered or masked during the fixation and embedding processes.

The article "Mechanism of Zuogui pill enhancing ovarian function and skin elastic repair in premature aging rats based on artificial intelligence medical image analysis" was retracted in 2025. Reasons: compromised peer review; a compromised editor; unreliable results or conclusions; concerns about the results or conclusions.

To optimize the immunohistochemical staining procedure and ensure accurate visualization of specific antigens, several additional steps were undertaken after the tissue sections underwent antigen retrieval. Firstly, to neutralize the activity of endogenous peroxidase that may interfere with the subsequent staining process, the tissue sections were treated with a 3% hydrogen peroxide solution for 10 min. This step effectively blocked the endogenous peroxidase activity, minimizing non‐specific background staining. The overnight incubation allowed for the primary antibodies to selectively bind to the target antigens within the tissue sections, enabling the subsequent detection and visualization of these specific proteins. After the overnight incubation, the tissue sections were rinsed with PBS to remove any unbound primary antibodies. To facilitate the detection of the primary antibodies, secondary antibodies were applied to the tissue sections and allowed to incubate for 10 min. Secondary antibodies, conjugated with specific markers or enzymes, bind to the primary antibodies, amplifying the signal and aiding in the subsequent visualization step. To enhance the visualization of the bound secondary antibodies, horseradish peroxidase was applied to the tissue sections and allowed to incubate at room temperature for 10 min. This enzyme catalyzes a chromogenic reaction that produces a distinct color, aiding in the localization and visualization of the target proteins. To visualize the final result, the tissue sections were treated with 3,3′‐diaminobenzidine (DAB), which interacts with the horseradish peroxidase to generate a brown staining signal specifically at the sites where the target antigens are located. Hematoxylin staining was then applied to the tissue sections to provide a contrasting blue counterstain, aiding in the examination of the tissue architecture. Following the staining process, the tissue sections were rinsed with tap water for 10 min to remove any excess staining reagents. Subsequently, the sections underwent dehydration by sequentially immersing them in a series of ethanol solutions of increasing concentration. This step ensured the removal of water and preservation of the stained tissue sections. To render the tissue sections transparent and facilitate the mounting process, xylene was applied to the sections. The xylene effectively removed the ethanol from the tissue, making it suitable for mounting. Excess xylene was gently removed using filter paper, and the sections were then sealed with neutral gum to protect the stained tissue sections and preserve them for subsequent analysis and examination.

### 2.5 Western blot (WB)

The remaining half of the surgically excised ovaries, intended for Western blot (WB) analysis, were cautiously preserved at a temperature of −80°C until further analysis could be carried out. The frozen ovarian tissues were maintained at this ultra‐low temperature, which facilitated the long‐term storage of biological samples without compromising their cellular integrity or protein composition. To quantitatively assess the levels of specific proteins of interest, including PI3K, Akt, mTOR, p‐PI3K, p‐Akt, p‐mTOR, Bcl‐2, Bax, and caspase‐3, in the ovarian tissue, a Western blot analysis was conducted. This widely employed technique allowed for the detection and quantification of target proteins within complex biological samples such as the ovaries. Prior to the protein extraction process, the stored ovarian tissues were homogenized using a specialized lysis buffer called RIPA buffer, which facilitated the disruption of cells and the release of proteins while preserving their native conformation. To prevent protein degradation during the extraction, protease inhibitor phenylmethylsulfonyl fluoride (PMSF) was added to the RIPA buffer. The homogenization was meticulously carried out, ensuring the complete disruption of cells and maximizing protein recovery. Following homogenization, the ovarian tissue and lysis buffer mixture were incubated on ice for 30 min. This step allowed for the complete solubilization of proteins and the preservation of their activity despite sub‐zero temperatures. To obtain the protein extracts, the homogenized samples were subjected to centrifugation at 12 000 rotations per minute (rpm) and a temperature of 4°C for 15 min. The centrifugation process effectively separated the insoluble cellular debris from the soluble supernatant, which contained the protein fractions of interest. The supernatants, carefully collected without disturbing the pellet, were then subjected to further analysis for protein quantification. The concentration of the extracted proteins in the supernatants was determined using a BCA (bicinchoninic acid) protein assay kit. This colorimetric assay measured the protein concentration in the samples by assessing the formation of a copper‐protein chelate complex. Through a series of chemical reactions, the amount of protein present in each sample was quantified, enabling accurate normalization and comparison of protein levels across multiple samples. The choice of voltage during the electrophoresis process (ranging between 80 and 120 V) depended on the specific gel system and the desired separation resolution. This transfer process, known as blotting, facilitated the immobilization of the separated proteins onto a solid support for subsequent antibody‐based detection. The PVDF membranes, known for their high protein‐binding capacity and compatibility with various detection methods, allowed for efficient transfer and retention of proteins.

The article "Mechanism of Zuogui pill enhancing ovarian function and skin elastic repair in premature aging rats based on artificial intelligence medical image analysis" was retracted in 2025. Reasons: compromised peer review; a compromised editor; unreliable results or conclusions; concerns about the results or conclusions.

To ensure accurate and specific protein detection, the PVDF membranes containing the transferred proteins were subjected to a blocking step. This step involved incubating the membranes with 5% nonfat dry milk at room temperature for a duration of 1 h. The nonfat dry milk acted as a blocking agent, effectively preventing non‐specific binding of antibodies and reducing background signal during subsequent antibody incubations. The overnight incubation allowed for the specific binding of the primary antibodies to their respective target proteins within the protein samples. After the overnight incubation, the PVDF membranes were rinsed to remove any unbound primary antibodies, and the corresponding secondary antibodies were applied. These secondary antibodies, conjugated with specific markers or enzymes, recognize and bind to the primary antibodies that had already bound to their respective target proteins. This secondary antibody binding further amplifies the signal and facilitates the subsequent detection of the target proteins. The membranes were then incubated at room temperature for 2 h to allow sufficient time for the secondary antibodies to bind to the primary antibodies. This incubation period ensured the effective visualization of the target proteins through the subsequent detection step. To visualize the protein bands, an enhanced chemiluminescence (ECL) reagent was used. This sensitive detection method utilizes a chemical reaction between enzymes linked to the secondary antibodies and the ECL reagent, resulting in the emission of light. The emitted light can then be captured using specialized imaging equipment, allowing for the visualization and quantification of the protein bands. For accurate quantification, an internal loading control, β‐actin, was used. β‐actin is a commonly used housekeeping protein, known for its stable expression across different tissue types and conditions. It serves as a reference point to normalize the grayscale intensity of the protein bands, facilitating the comparison of protein levels across different samples. After the protein bands were developed using the ECL reagent, the grayscale intensity of the bands was determined using Image‐Pro Plus 6.0 software, enabling quantitative analysis of the protein expression levels within the ovarian tissue samples.

### 2.6 TUNEL

TUNEL assay was carried out in line with the manufacturer's protocols. Ovarian tissues were sunk in 4% paraformaldehyde solution overnight, dehydrated, and subsequently embedded in paraffin, before being cut into sections of 4 μm thickness and placed on a numbered glass slide covered with polylysine. Slices of dewaxed tissue were incubated with proteinase K (20 mg/mL) in a moist environment for 15 min, and the activity of endogenous peroxidase was suppressed after treated with 3% H_2_O_2_ for 10 min. Following this, slices were kept in a damp chamber and processed with a 37°C TdT labeling buffer for 1 h. DAPI served as a counterstain. Positive cells appeared green, while the nuclei were colored with DAPI to determine the character of the cells.

The article "Mechanism of Zuogui pill enhancing ovarian function and skin elastic repair in premature aging rats based on artificial intelligence medical image analysis" was retracted in 2025. Reasons: compromised peer review; a compromised editor; unreliable results or conclusions; concerns about the results or conclusions.

### 2.7 Statistical analysis

For the statistical analysis, we utilized the GraphPad 8.0 software, a widely used tool in scientific research. The measurement data generated in our study were presented in a descriptive manner, specifically as means accompanied by the corresponding standard deviation (SD) values. To determine the significance of differences among the five groups, we applied a statistical test known as one‐way analysis of variance (ANOVA). However, this analysis was performed exclusively if the criteria for normal distribution and homogeneity of variance were met by the univariate quantitative group data. To make comparisons between specific groups, we employed Student's *t*‐test, a statistical test commonly used for examining the significance of differences between two groups. In our study, statistics were considered significant when the calculated *p*‐value was less than 0.05, indicating statistical significance at a 95% confidence level. Through this rigorous statistical analysis approach, we aimed to provide robust and reliable results to support the conclusions drawn from our research findings.

## 3 RESULTS

### 3.1 ZGP regulated serum MDA and SOD in POI rats

An improvement in the MDA levels and an increase in SOD levels in response to ZGP treatment were observed, and this effect showed a dose‐dependent relationship (all *p* < 0.001, Figure 1).

**FIGURE 1:** ZGP inhibited MDA and increased SOD in plasma. (A) The result of ELISA showed that the rise of MDA was blunted in the POI model by ZGP. (B) The result of ELISA showed that the reduction of SOD was reversed by ZGP. Compared with the blank group, ***p < 0.001. Compared with the model control group, ###*p *< 0.001.

### 3.2 ZGP reduced apoptotic GCs in the antral follicles

To understand the apoptosis of GCs, TUNEL assay was undertaken on ovarian sections. Green fluorescence represents apoptotic cells. As shown in Figure 2, few TUNEL positivity was captured in the blank group, however in POI mice widespread TUNEL positive staining was seen in GCs. Following ZGP treatment, GCs apoptosis in the antral follicles descended in ZGP‐treated groups with a dose‐dependent tendency.

**FIGURE 2:** Granulosa cells (GCs) apoptosis in the antral follicles was visualized. TUNEL immunofluorescence staining of the ovaries of GCs. Green represented TUNEL‐positive signal. ZGP inhibited the apoptosis in POI rats and the effect was enhanced with the increasing dose. Magnification is ×400.

The article "Mechanism of Zuogui pill enhancing ovarian function and skin elastic repair in premature aging rats based on artificial intelligence medical image analysis" was retracted in 2025. Reasons: compromised peer review; a compromised editor; unreliable results or conclusions; concerns about the results or conclusions.

### 3.3 ZGP increased the expression of p‐PI3K, p‐Akt, and p‐mTOR in ovarian tissue

As Figure 3 indicated, the expressions of the three proteins were all relatively absent in the model control group against that in the blank one, especially in GCs. By comparison, recovered levels of p‐PI3K, p‐Akt, and p‐mTOR in all ZGP‐treated groups at any dose were observed and the tendency of dose‐dependency was also clear.

**FIGURE 3:** ZGP activated the expression of p‐PI3K, p‐Akt, and p‐mTOR. Brown representing the immunohistochemistry‐positive signal. The diminution of three proteins in POI could be overturned by ZGP with a dose‐dependent tendency. Magnification is ×400.

### 3.4 ZGP increased the expressions of p‐PI3K, p‐Akt, p‐mTOR, and Bcl‐2 and suppressed the expressions of Bax and caspase‐3 in ovarian tissue

For the purpose of further exploration of the mechanism of ZGP in POI treatment, protein expression linked to PI3K/Akt/mTOR signaling pathway and apoptosis‐related proteins was assayed by WB. Figure 4 demonstrated that expressions of PI3K, Akt, and mTOR did not differ significantly between groups (all *p *> 0.05). After ZGP treatment, the disadvantageous responses were countered and better effects were observed in the higher dose. Relative to the model control group, ZGP promoted the level of Bcl‐2 and the effect notably excluding the low dose group (*p *> 0.05, *p *< 0.05, and *p *< 0.01, respectively, Figure 4). The findings manifested that the inhibition of PI3K/Akt/mTOR signaling pathway and apoptosis occurred in the POI rats while ZGP alleviated the negative influences with a tendency of dose‐dependency.

**FIGURE 4:** ZGP activated PI3K/Akt/mTOR signaling pathway and inhibited apoptosis. Western blot showed expressions of p‐PI3K, PI3K, p‐Akt, Akt, p‐mTOR, mTOR, Bcl‐2, Bax, and caspase‐3. Compared with the blank group, ***p < 0.001. Compared with the model control group, #*p *< 0.05, ##*p *< 0.01, and ###*p *< 0.001.

## 4 DISCUSSION

Premature aging is the phenomenon in which a person shows early signs of aging, either physically or mentally. In women, decreased ovarian function is one of the main causes of premature aging. The ovaries are an important part of the female reproductive system, responsible for producing eggs and hormones, and maintaining reproductive function and endocrine balance. When ovarian function is impaired, problems such as menstrual disorders, infertility, and abnormal sex hormone levels can occur. At present, the diagnosis and study of premature aging mainly rely on microscopic observation of tissue sections. However, traditional microscopy techniques have some limitations in terms of resolution and sample handling, limiting the detailed observation and analysis of cell and tissue structures. Therefore, optical microscope image detection, as a new technology, has been widely used in biomedical research. Optical microscopy image inspection can obtain high‐resolution tissue images through optical imaging techniques and provide more comprehensive and detailed information.

The article "Mechanism of Zuogui pill enhancing ovarian function and skin elastic repair in premature aging rats based on artificial intelligence medical image analysis" was retracted in 2025. Reasons: compromised peer review; a compromised editor; unreliable results or conclusions; concerns about the results or conclusions.

The dermis is located below the epidermis and is composed of collagen fibers, elastic fibers, glucosamine, and other tissues. The dermis is divided into papillary dermis and reticular dermis, and there is no clear boundary between the two. Papillary dermal fibers are thin and zigzag with the epidermis, while reticular dermal fibers are thicker and thicker. Subcutaneous tissue is located below the dermis and consists of lobules of fat cells and connective tissue compartments. The subcutaneous tissue has a thermal insulation and buffering function that protects the body from trauma and stores nutritious energy. The main function of the skin is to protect the human body from the external pathogenic environment, and to resist harmful stimuli such as microorganisms, pathogenic bacteria, and radiation. In addition, it can also reduce the shear force on the skin, prevent the loss of water and electrolytes, and maintain a stable body temperature.

With the growth of age, the impact of the daily environment, and long‐term bad habits, the elasticity of the skin gradually decreases, and the problems of wrinkles, relaxation, and loss of elasticity appear. Lack of moisture in the skin can lead to dry skin and loss of elasticity. Therefore, we should drink plenty of water, use moisturizing products, and avoid prolonged exposure to dry environments. Eating foods rich in vitamins C and E can promote collagen synthesis, which increases the elasticity of the skin. Eating enough protein and healthy fats also helps maintain the elasticity and health of your skin. Gentle cleansing and exfoliation can help remove dead skin cells from the surface of the skin and promote cell renewal. Using skin care products that contain antioxidants and promote collagen production can help improve the elasticity of your skin. Getting moderate exercise can improve blood circulation, increase the supply of nutrients to the skin, and help repair damaged skin tissue. At the same time, avoiding excessive exposure to UV rays and harmful substances is also key to maintaining healthy and resilient skin.

The article "Mechanism of Zuogui pill enhancing ovarian function and skin elastic repair in premature aging rats based on artificial intelligence medical image analysis" was retracted in 2025. Reasons: compromised peer review; a compromised editor; unreliable results or conclusions; concerns about the results or conclusions.

Existing studies have shown that Zuogui pill can improve ovarian function and has the potential to delay premature aging. Through optical microscope image detection technology, we can observe and analyze the changes of cell structure and tissue morphology of ovaries in rats with premature aging. By processing and analyzing the images, quantitative information about ovarian function, such as ovarian size, follicle quantity and quality, was obtained. The effect of Zuogui pill on ovarian function was evaluated by comparing the image data of Zuogui pill group and control group. Optical microscopy image detection technology can also help us observe changes in ovarian blood vessels. Blood vessel supply is essential for maintaining ovarian function, and vascular degeneration is an important feature of premature aging. Through optical microscope image detection technology, the changes of blood vessel density and blood vessel morphology were observed and analyzed, so as to further understand the effect of Zuogui pill on blood vessel reconstruction and functional improvement.

The present study observed the rise of serum MDA and the decline of SOD in POI rats, which could be ameliorate by ZGP with a dose‐dependency. The expression of apoptosis of GCs enhanced after cisplatin induced and was ameliorated by ZGP. Furthermore, the inhibition of PI3K/Akt/mTOR signaling pathway in POI was found, and the activation of the pathway occurred after ZGP treatment. The findings demonstrated the protective effects of ZGP on POI through relieving oxidative stress and preventing GCs apoptosis, and the underlying principle might be the activation of PI3K/Akt/mTOR signaling pathway, proving ZGP perhaps a promising agent against POI.

Primordial follicles activation and the differentiation and proliferation of surrounding somatic and GCs are critical to the ovulation process. Nevertheless, premature activation would cause loss of dormant follicle reserves then bring about POI resulting in infertility. For POI, the main pathogenesis has not yet elaborated, the etiology unclear, and the treatment unsatisfactory.^10^ The formula of TCM ZGP originates from a well‐known ancient prescription of the Ming Dynasty. The uniqueness of ZGP has been noticed in treatment of some miscellaneous diseases such as POI, diabetes, asthma, and osteoporosis.^11^ Clinical and experimental results showed that ZGP had good efficacy in treating POI, whether alone or in combination.^12^, ^13^, ^14^, ^15^ However, there are few related in‐depth studies and pharmacological mechanisms of ZGP for POI are not yet distinct.

Oxidative stress participates in the POI, which promotes lipid peroxidation, damages proteins and DNA, and causes apoptosis.^16^, ^17^, ^18^ MDA, a byproduct of oxidative stress, and SOD, an essential antioxidant defense enzyme, are routinely employed as oxidative damage markers to identify the extent of oxidative damage and protective responses respectively.^19^ Bu Shen Huo Xue Tang, another TCM formula, is clinically employed to treat POI. It owned the effect of increasing SOD and reducing MDA on autoimmune POI in mice and the major ingredient is *Rehmannia glutinosa libosch*.^20^ *Radix Rehmanniae* polysaccharides could enhance SOD and reduce skin MDA in mice treated with ultraviolet B ray.^21^ As we known, one of the major components in ZGP is *Rehmanniae radix praeparata*. Hence, we assumed that ZGP could also reduce the serum MDA and raise SOD. The results were consistent with our hypothesis, demonstrating oxidative stress existed in POI model, and ZGP could alleviate it with a dose‐dependency.

The article "Mechanism of Zuogui pill enhancing ovarian function and skin elastic repair in premature aging rats based on artificial intelligence medical image analysis" was retracted in 2025. Reasons: compromised peer review; a compromised editor; unreliable results or conclusions; concerns about the results or conclusions.

Optical microscope image detection is a valuable technique to study the mechanism of Zuogui pill to enhance ovarian function in rats with premature aging. In previous studies, oxidative stress has been found to play an important role in the occurrence and development of premature aging. Oxidative stress can cause lipid peroxidation, protein and DNA damage, and promote cell apoptosis. Therefore, we have reason to believe that oxidative stress may also be involved in the effect of Zuogui pill on the enhancement of ovarian function in rats with premature aging. In this study, we used optical microscopy image detection techniques to observe and analyze changes in oxidative stress levels in ovarian tissue of premature aging rats. We assessed the extent of oxidative stress by detecting markers of oxidative damage, such as malondialdehyde (MDA) and superoxide dismutase (SOD). MDA is a by‐product of oxidative stress, while SOD is an important antioxidant defense enzyme. By comparing and analyzing the ovarian tissue of Zuogui pill group and control group, we can reveal the regulation effect of Zuogui pill on oxidative stress. Our results support our hypothesis. We observed a significant oxidative stress response in the premature aging rat model, manifested by increased serum MDA levels and decreased SOD activity. However, after treatment with Zuogui pill, we observed a trend of decreasing serum MDA level and increasing SOD activity. This suggests that Zuogui pill can alleviate oxidative stress in ovaries of premature aging rats in a dose‐dependent manner.

Apoptosis is deemed to be the essential mechanism of cell death involving the depletion of oocytes during growth from primordial to antral follicles.^22^ As noted earlier, apoptosis could result from oxidative stress. It is also widely recognized that Bcl‐2 protein family like anti‐apoptotic Bcl‐2 and pro‐apoptotic Bax regulates follicular growth/atresia. Meanwhile, Bcl‐2 precludes caspase apoptosis protein from activation.^22^, ^23^, ^24^, ^25^ Caspase‐3, a vital determinant of apoptosis, whose activation causes DNA damage and cell apoptosis.^26^ Regulating the Bax/cytc/caspase‐3 pathway could advance ovarian reserve function by maintaining a balance between Bax and Bcl‐2. Generally, the TCMs that improved POI could raise Bcl‐2 and lower Bax and caspase‐3 in the ovary, reducing GCs apoptosis. Therefore, in POI model control group, we observed the occurrence of GCs apoptosis, and the levels of apoptosis‐related proteins altered with up‐regulated Bax and caspase‐3 and down‐regulated Bcl‐2. The disadvantageous alterations would be countered by ZGP. According evidence above, we inferred that ZGP perhaps exerted a significant protective efficacy on GCs against apoptosis by restraining oxidative stress.

The article "Mechanism of Zuogui pill enhancing ovarian function and skin elastic repair in premature aging rats based on artificial intelligence medical image analysis" was retracted in 2025. Reasons: compromised peer review; a compromised editor; unreliable results or conclusions; concerns about the results or conclusions.

The process of apoptosis is not only the consequence of oxidative stress, but the PI3K/Akt/mTOR signaling pathway participated in studies.^27^, ^28^ Studies had confirmed that the PI3K/Akt/mTOR signaling pathway was tied to oocyte growth and regulation, and impacted on primary follicle survival and development, promoting proliferation and differentiation of GCs and preventing its apoptosis as well.^29^ Once PI3K is activated, it produces phosphatidylinositol (PIP3) and results in transcription of Akt. Subsequently, a cascade of signal transduction pathways occurred. The inhibitory system is crucial for primordial follicles to maintain a quiescent state and avoid POI.^30^ A network analysis identified Zuogui Yin, a TCM with the same origin as ZGP that may act as a therapeutic method in male infertility by regulating six pathways, including the PI3K‐Akt signaling pathway.

Although our work uncovered a possible mechanism of ZGP for POI treatment, there were still some shortcomings in the experiment. The sample scale was not large enough. What is the specific mechanism of ZGP regulating PI3K/AKT/mTOR signaling pathway has yet to be explored further. In addition, a common problem with TCM compounds is that it is not clear which ingredient is at work. We will refine these flaws in future experiments.

## 5 CONCLUSIONS

Through the processing and analysis of medical images, artificial intelligence can provide accurate diagnosis and prediction, and provide more comprehensive auxiliary decision support for clinicians. In this study, we used artificial intelligence medical image analysis technology to evaluate ovarian tissue, helping us to understand the mechanism of the Zuogui pill's enhancement of ovarian function in premature aging rats. This shows the potential of AI medical image analysis in studying and improving reproductive health. This study discussed the role of artificial intelligence medical image analysis in skin elastic repair. Through the image analysis of the skin tissue, we can accurately assess the elastic state of the skin and provide a personalized skin elastic repair program based on the evaluation results. The results showed that the optical microscope image detection revealed the mechanism of Zuogui pill on enhancing ovarian function in rats with premature aging. Zuogui pill treatment group showed a trend of decreasing apoptosis. Apoptosis is an important mechanism in follicle growth/atresia, and oxidative stress is a key factor in apoptosis. Zuogui pill may reduce the apoptosis of ovarian cells by inhibiting oxidative stress response, thus improving ovarian function. Zuogui pill treatment group showed a trend of regulating the Bax/cytc/caspase‐3 pathway. The levels of Bax protein and caspase‐3 are indicators of apoptosis, whereas Bcl‐2 acts as an inhibitor of caspase‐3 activation, thereby reducing apoptosis. By maintaining the balance between Bax and Bcl‐2, Zuogui pills have the potential to promote the improvement of ovarian reserve function. ZGP could enhance the function of the ovary by relieving oxidative stress and activating the PI3K/AKT/mTOR pathway to reverse the GCs apoptosis in the POI rat model. The mechanism for ZGP to treat POI was revealed at the molecular level in our work, providing a theoretical basis for clinical practice.

The article "Mechanism of Zuogui pill enhancing ovarian function and skin elastic repair in premature aging rats based on artificial intelligence medical image analysis" was retracted in 2025. Reasons: compromised peer review; a compromised editor; unreliable results or conclusions; concerns about the results or conclusions.

## CONFLICT OF INTEREST STATEMENT

The authors declare no competing interests.

## Data Availability

Data will be made available on request.
